# Effect Evaluation of Electronic Health PDCA Nursing in Treatment of Childhood Asthma with Artificial Intelligence

**DOI:** 10.1155/2022/2005196

**Published:** 2022-03-28

**Authors:** Wensong Li, Zhidong Liu, Tao Song, Chunlong Zhang, Jianzhen Xue

**Affiliations:** Department of Pediatrics, Qingdao Jiaozhou Central Hospital, No. 99, Yunxi Henan Road, Jiaozhou, Shandong Province, 266300, China

## Abstract

Asthma in children has a long duration and is prone to recurring attacks. Children will feel chest tightness, shortness of breath, cough, and difficulty breathing when they are onset, which has a serious impact on their health. Clinical nursing is of great significance in the treatment of childhood asthma. At present, the electronic health PDCA nursing model is widely used in clinical nursing as a common and effective nursing method. Therefore, it is very important to evaluate the efficacy of the PDCA nursing model in the treatment of childhood asthma. With the development of artificial intelligence, artificial intelligence can be used to evaluate the effect of the PDCA nursing model in the treatment of childhood asthma. The BP network can effectively perform data training and discrimination, but its training efficiency is low, and it is easily affected by initial weights and thresholds. Aiming at this defect, this work uses the genetic simulated annealing (GSA) algorithm to improve it. In view of the problems that the genetic algorithm falls into local minimum and simulated annealing algorithm has a slow convergence speed, the improved genetic simulated annealing algorithm is used to optimize the BP neural network, and an improved genetic simulated annealing BP network (IGSA-BP) is proposed. The algorithm not only reduces the problem that the BP network has an influence on initial weight and threshold on the algorithm but also improves the population diversity and avoids falling into local optimum by improving the crossover and mutation probability formula and improving Metropolis criterion. The proposed method has more efficient performance.

## 1. Introduction

Asthma is a heterogeneous disease characterized by chronic airway inflammation and airway hyper-responsiveness. The main clinical manifestations are wheezing, coughing, shortness of breath, and chest tightness, which often occur or intensify at night and in the early morning, and are recurrent. The specific presentation and severity of respiratory symptoms can vary over time and are often accompanied by variable expiratory airflow limitation. Symptoms such as chest tightness, difficulty breathing, and coughing during an asthma attack can cause physical discomfort in children, which in turn can cause psychological panic, anxiety, and tension. Asthma in children is a common respiratory disease in children. Due to repeated attacks, it is difficult to cure completely, which seriously affects the physical and mental health of children and also brings serious economic burden and mental pressure to the parents of children [1–4].

In recent years, with the changes in people's production and living environment and many other aspects, the prevalence of various allergic diseases, including asthma, has shown a significant upward trend in the world. Epidemiological survey data show that the prevalence of asthma in urban Chinese children under 14 years old was 1.09% in 1990, 1.97% in 2000, and 3.02% in 2010. The results of the 3 childhood asthma prevalence surveys conducted in China show that the prevalence of childhood asthma in China is increasing year by year. In the past 10 years, the prevalence of childhood asthma has increased by 64.84%, mainly in the age group of 6 to 14 years old, with a prevalence of 3.4% [5–8].

A series of symptoms such as coughing, chest tightness, and difficulty breathing may occur due to an asthma attack. With the onset of asthma, there will be respiratory distress, sense of impending death, sleep disturbance at night, and other effects. The occurrence of these symptoms will also cause children to have certain emotional disorders such as fear, anxiety, and depression, which will seriously affect the quality of life of children. Affected by the condition of asthma, the incidence of behavioral problems in children with asthma is higher than that in other normal children. Because children are currently in a period of rapid growth and development, their cognitive abilities and personality psychology are still under development, and their ability to withstand external stress is poor. At the same time, due to the attack of asthma, the children cannot concentrate on study and exercise like normal children, and the psychological burden is heavier. The long-term adverse stimuli produced by asthma have a profound impact on the development of children's psychosocial functions [9–12].

The PDCA cycle theory has now become the basic method of nursing management. The basic method of its operation is to manage the cycle through the scientific work procedures of plan, do, check, and action. The starting points are all higher than the previous cycle. PDCA cycle theory, as a scientific work procedure to carry out quality management activities, has been widely used in enterprise management and has achieved remarkable results. It is one of the effective management methods recognized by the management field, has been widely used in various fields, has achieved remarkable results, and has been increasingly concerned and valued by nursing managers. A large amount of literature shows that many nursing managers have widely introduced PDCA cycle theory into nursing quality management and teaching and clinical practices and have produced many theoretical and practical results. The 2014 edition of GINA pointed out that the long-term management of asthma is crucial to the effect and prognosis of asthma treatment and re-emphasized that long-term management should be integrated throughout the asthma cycle management [13–15].

For this reason, it has become a very important issue to evaluate the therapeutic effect of the PDCA nursing model in children with asthma. With the development of artificial intelligence, more and more research combine medical treatment with artificial intelligence. This work combines artificial intelligence with this subject and proposes an improved genetic simulated annealing BP network to evaluate the therapeutic effect of the PDCA nursing model applied to children with asthma.

The main contribution of this study is as follows:

- The issues that the BP network's findings are easily influenced by initial values and criteria, and resolution is sluggish and prone to local optimization, this work attempts to improve the BP network using GA and SA. Therefore, the effectiveness of the electronic health PDCA nursing model in the treatment of asthma in children was assessed.
- Create an IGSA algorithm by analyzing and summarizing the principles of GA and SA algorithms, as well as their relative benefits and drawbacks. Adaptive modification in biological operations can improve algorithm resolution time by increasing crossover and mutation frequency. The optimization algorithm capability is increased by enhancing the Metropolis requirement.

The rest of the study is organized as the related work of the study is discussed in Section 2. In Section 3, the proposed method is presented.  Section 4 examined the experimental results.  Section 5 illustrated the conclusion.

## 2. Related Work

Since the 1980s, the management method of PDCA cycle theory began to enter the medical field, and after popularization and application, it has gradually become a management tool widely recognized by the industry. In recent years, the use of PDCA cycle theory abroad has been relatively mature, and good results have been achieved in nursing quality management and other work. Reference [16] used the PDCA cycle to carry out nursing staff education in the hospital, and the satisfaction of nursing staff was significantly improved. Reference [17] used PDCA cycling to improve blood glucose testing in hospitalized patients and contributed to the improvement of quality of care. Reference [18] carried out the application of PDCA circulation in the ICU, which greatly reduced the rate of catheter-related blood infection. Literature [19] applied the FOCUS-PDCA theory to solve clinical nursing problems and confirmed that FOCUS-PDCA can solve multifaceted and complex clinical nursing quality problems and is a systematic, logical, and accurate management method. Literature [20] applied PDCA cycle theory in the nursing of severe traumatic brain injury and achieved positive results.

In recent years, the application of PDCA cycle theory to nursing quality management, health education, and chronic disease management has achieved good results in the domestic nursing field. Literature [21] carried out a diabetes-health-education-research on the PDCA cycle combined with the whole diabetes health education form, that is, nursing problems-self-learning-treatment goals, and achieved remarkable results. Reference [22] applied the PDCA cycle combined with the PIO follow-up management project in the management of T2DM patients with NAFLD, which effectively improved the patients' self-care behavior and quality of life. Literature [23] applied the PDCA cycle to carry out postoperative rehabilitation health education for patients with minimally invasive lumbar spine surgery, which effectively improved patients' awareness of rehabilitation knowledge and improved their motor function. Literature [24] implemented PDCA cycle health education to effectively mobilize the enthusiasm of children and parents and to achieve the control of childhood asthma. Literature [25] implemented the PDCA cycle nursing model for patients with myocardial infarction, which improved the patients' quality of life and satisfaction and reduced the number of angina pectoris attacks. Reference [26] implemented nursing intervention based on the PDCA cycle model, which reduced the postoperative bleeding volume and the incidence of infection in patients with dangerous placenta previa and improved the quality of life of the patients. Reference [27] applied the PDCA cycle mode to implement health education for the normal high-blood pressure occupational population, so that the blood pressure level of the target population was effectively controlled and the lifestyle tended to change positively. It can effectively prevent hypertension and its complications in the occupational population. Literature [28] obtained satisfactory results by using the PDCA cycle management model in the implementation of gastroenterology health education. Literature [29] used the PDCA cycle in oral and gynecology clinical teaching, respectively, and achieved good results. Literature [30] applied the PDCA cycle theory in the process of nursing record quality management, which effectively improved the quality of medical record writing. Literature [31] used the PDCA cycle for emergency department nursing quality management. Literature [32] used the PDCA cycle for oral diagnosis and nursing management and achieved good results, improving nursing quality and patient satisfaction Table 1.

## 3. Method

In this work, the genetic algorithm and the simulated annealing algorithm are combined and improved first, and then the improved algorithm is combined with the BP network. Finally, an artificial intelligence-based model was designed to evaluate the effect of the electronic health PDCA care model in the treatment of childhood asthma.

### 3.1. BP Network

The BP (backpropagation) network was proposed by researchers such as Rumelhart and McClelland in 1986. It is a multilayer feedforward neural network trained by forwarding the propagation of errors. Through the forward propagation of the data, an error is generated in the comparison with the expected output. The error is then propagated back to each node, and the weights and thresholds of each node are continuously revised. Then, the error is decreased along the gradient, and the target output is continuously approached to achieve the optimal network structure. The structure of the BP network is shown in Figure 1.

The structure of the ordinary three-layer BP network is divided as follows: the first layer of input layer, the second layer of hidden layer, and the third layer of output layer. The learning steps of the BP network can be summarized as follows.

Step 1: *Initialization*. Initialize the neural network structure, set the target accuracy *E*, set the maximum number of iterations *M*, and set the initial weights and thresholds or directly use random real numbers instead.
Step 2: *Forward Propagation*. Suppose the BP algorithm has *n* groups of training sets (*x*_1_, *x*_2_,…, *x*_*n*_), then there are also *n* groups of expected output values (*y*_1_, *y*_2_,…, *y*_*n*_). At the same time, the number of nodes in each layer of the BP neural network is set as (*n*_1_, *n*_2_, *n*_3_). When the *a*-th sample of the training set is input, according to the neural network, the forward propagation formula is calculated as follows:
  (1) $$\begin{array}{c} h_{p}^{a}=\sum_{i=1}^{n_{1}}w_{ip}x_{i}^{a},\\ y_{k}^{a}=\sum_{p=1}^{n_{2}}w_{pk}h_{p}^{a}, \end{array}$$
where *h*_*p*_^*a*^ is the output of the *p*-th neuron in the hidden layer and *y*_*k*_^*a*^ is the output of the *k*-th neuron in the output layer. *w*_*ip*_ is the connection weight between the input layer and the hidden layer and *w*_*pk*_ is the connection weight from the hidden layer to the output layer.
Step 3: *Error Calculation*. The BP network takes the minimum mean square error as the criterion and backpropagates the error to adjust the weights. The error caused by the output to the output result and the expected output result of the training set when the BP network process is completed in a single time is shown in the following equation:
  (2) $$\begin{array}{c} E_{a}=0.5\sum_{k=1}^{n}{\left(c_{k}^{a}-y_{k}^{a}\right)}^{2}, \end{array}$$
where *c*_*k*_^*a*^ is the expected output and *y*_*k*_^*a*^ is the actual output value.
Step 4: *Error Backpropagation to Correct Weights and Bias*. The calculated error is returned to each corresponding neuron layer by layer for correction. The correction value for each layer is as follows:
  (3) $$\begin{array}{c} \Delta w=-\eta \frac{\partial E_{a}}{\partial w},\\ \Delta b=-\eta \frac{\partial E_{a}}{\partial b}. \end{array}$$
Step 5: *Error Accuracy and End Judgment*. Judging and comparing the training output results with the expected results and the error accuracy set by the initialization, that is, for any training set sample and its output results, it satisfies the following equation:

(4) $$\begin{array}{c} \left|c-y\right|<\varepsilon , \end{array}$$

where *ε* is the set network training expected error accuracy.

If each training sample in the network training process meets the error requirements of the above formula, then the BP network training is completed, or the network training times have reached the maximum training algebra; otherwise, return to Step 2 to continue network training.

There are still many problems in the practical application of traditional BP neural networks. (1) The BP network algorithm is an error gradient descent algorithm that approaches the ideal value with continuous correction. However, when the training objective function mapping structure is complex, the training efficiency is reduced. (2) Since the training objective function often has a certain complexity, in the process of training, some neuron output results in multigeneration training may be too close to the expected value, which will make the error of these neurons extremely small, resulting in a flat error iteration. In the region, the weight error hardly changes, which in turn leads to low training efficiency. (3) The algorithm structure of the BP network makes the network easy to fall into the local optimum during training, while ignoring other global optimum values, making the training result unsatisfactory. (4) The initial weights and thresholds of the BP network neurons have a decisive effect on the subsequent network training. A good initialization will enable the neural network to learn efficiently and quickly and maximize the global optimization ability. The initialization with excessive deviation will make the network training process very slow, and the system may need several iterations to gradually complete the training. (5) The training of the BP network is a step-by-step process. With the continuous training, the network learning and prediction ability is also continuously improved. However, this trend also has certain limitations. After exceeding it, the learning and prediction ability of the network decreases as the training progresses.

This study is dedicated to using genetic algorithms and simulated annealing algorithms to optimize the BP network to enhance the global search ability and training speed. This avoids the problems of overfitting and local convergence and improves the capabilities of the BP network as a whole.

### 3.2. Genetic Algorithm

The genetic algorithm transforms complex and abstract optimization problems into simple and specific steps of chromosomal gene crossover, mutation, and selection in biological genetic evolution through mathematical principles, and it has good algorithm convergence and optimization capabilities. The general flow of the genetic algorithm is shown in Figure 2.

The main calculation steps of the genetic algorithm are as follows: (1) Chromosome coding the optimized data to make data that can be genetically processed. (2) Initialize the population and its parameters, set the maximum genetic algebra, decide the stop timing, etc. (3) Calculate the fitness value of all individuals to the objective function, which determines the quality of the individual in the population. (4) Selection, according to the individual fitness value, the population is selected and screened, and the better individual is selected to enter the next generation. (5) Crossover, the crossover operation is performed on the chromosome encoding of the individual. (6) Variation, mutating the individual chromosome code. (7) Update individual chromosomes to generate new populations. (8) Judge the termination conditions, and return to Step 3 if the requirements are not met. (9) Output the chromosome of the optimal individual in the population of the final result, and decode to obtain the optimal solution of the objective function.

Coding is the foundation of genetic algorithm, and the appropriate coding method can determine the efficiency and accuracy of the optimization algorithm. When encoding data, it is necessary to preserve the characteristics of the original data as much as possible and to simplify its structure as much as possible. An unreasonable coding method may lead to individuals without feasible solutions in the feasible solution set of the optimization algorithm or being unable to find the optimal target in the genetic process.

The main function of the population is to provide evolutionary sites and search ranges for heredity, and a good population should contain all possible solutions to the problem. Initializing the population usually affects the various algorithm capabilities of the genetic algorithm. In practical applications, a population is usually generated in a random manner or a population is randomly generated under a certain constraint. In the subsequent steps, the chromosomes of the individuals of the population are used as genetic operators to initialize the population as the starting point, and the optimal solution is output through iterative operations.

Fitness function is the only standard to measure the quality of individuals in a population. This enables the genetic algorithm to perform global search optimization without any external factors. The establishment of fitness function directly affects the convergence efficiency of genetic algorithms.

Contrastive selection is one of the three key steps of the genetic algorithm. Its purpose is to compare and screen the parent and offspring individuals in the population. The individual with a higher fitness value wins and goes to the next step. According to the fitness value of each individual and other different criteria and algorithms, the selection operation preserves the individuals with better genetic codes to the next generation and eliminates some inferior individuals, so that the entire population evolves.

Crossover operation is one of the important parts of the genetic algorithm, which refers to the unexpected phenomena that occur in the process of chromosome division and replication in real cells. That is, during the replication process of two homologous chromosomes, parts of the same parts are exchanged, so that it is possible to produce two individuals different from the parent.

Mutation operation is one of the important parts of the genetic algorithm, which imitates the genetic mutation of biological genetic evolution in reality.

As a random search algorithm, the genetic algorithm has extremely efficient global optimization ability. The evolution process is carried out after encoding the target into a chromosome. The algorithm is not affected by the continuous-discrete characteristics and differentiable characteristics of the function and has a wider application range. Algorithmic search is more autonomous, only the fitness function is used as the criterion, and there is no dependence on other conditions. However, genetic algorithms also have flaws. When the fitness of a small number of individuals is significantly better than that of other individuals in the population, the size of the offspring of these individuals will gradually expand to occupy the majority of the population, making it more likely that similar genes will be passed on to the next generation. Individuals will be concentrated near the local optimum, causing the evolutionary direction of the population to tend to be fixed. The parameter setting is more dependent on empirical selection, and improper setting can easily lead to premature convergence to the local precocious problem. The discrete coding of chromosomes reduces the search ability of the genetic algorithm in the local area, resulting in wobbles. To sum up, genetic algorithms can improve each other by combining with other optimization algorithms.

### 3.3. Simulated Annealing Algorithm

The simulated annealing algorithm is a commonly used optimization algorithm, which usually follows the following steps.

Step 1: Set the initial temperature *T*_0_, annealing rate *λ*, number of iterations *N*, and termination temperature *T*, randomly generate an initial solution, and calculate the objective function value of the solution. Temperature is the basic framework of the simulated annealing algorithm, and the entire process runs between the initial and termination temperatures. The most commonly used annealing method is exponential descent:
  (5) $$\begin{array}{c} T\left(n+1\right)=\lambda T\left(n\right). \end{array}$$
The annealing rate *λ* is a positive number less than 1, usually between 0.8 and 0.99. If the value is too small, the annealing speed will be too fast, and the algorithm will end before convergence; if the value is too large, it is more likely to obtain a high-quality solution, but the amount of computation will increase accordingly.
Step 2: According to the generated disturbance function, the current solution is changed in the solution space, a new solution is generated, and the objective function value of the solution is calculated. The objective function measures the goodness of the understanding, similar to the fitness function in the genetic algorithm, and indicates the direction of continuous optimization in the simulated annealing algorithm.
Step 3: If the new solution is better than the old solution, replace the current solution with the new solution. Otherwise, according to the Metropolis criterion, accept the new solution with a certain probability to replace the current solution:
  (6) $$\begin{array}{c} P=\left\{\begin{array}{cc} \exp\left(\frac{E\left(n\right)-E\left(n-1\right)}{T\left(n\right)}\right), & E\left(n+1\right)<E\left(n\right),\\ 1, & \text{others}. \end{array}\right) \end{array}$$
When the temperature is high, the probability of accepting a poor new solution is high, which makes the simulated annealing algorithm have a high probability of jumping out of the local optimal solution at this stage. As the annealing progresses, this probability does not decrease, and eventually, only a better solution is approximated. Combined with the characteristics of the simulated annealing algorithm, it can be seen that the global search is emphasized in the high-temperature stage, and the local search is emphasized in the later low-temperature stage. So that the final solution converges to the optimal solution more efficiently.
Step 4: If the maximum number of iterations is reached, go to the next step. Otherwise, go back to Step 2.
Step 5: Perform an annealing operation, reduce the temperature, and reset the number of iterations.
Step 6: If the termination temperature is reached, the algorithm ends and the optimal solution is output. Otherwise, go back to Step 2.

The simulated annealing algorithm is relatively simple and easy to use, and it can still handle complex problems efficiently. The optimal solution has nothing to do with the initial solution. With the progress of annealing, ideally, the algorithm must converge to the global optimal solution. According to the screening of Metropolis criterion, the global search ability of simulated annealing algorithms is very good. However, the number of iterations of the algorithm is relatively large, which increases the amount of calculation. There is a contradiction between the annealing rate and the effect of the algorithm. Too fast annealing will lead to failure to converge to the optimal solution, and slow annealing operation will increase the calculation time of the algorithm, which requires the user's experience balance. In summary, the simulated annealing algorithm can be combined with other optimization algorithms to improve the overall performance.

### 3.4. Improved Genetic Simulated Annealing Algorithm

Genetic simulated annealing algorithm is a combination of genetic algorithm and simulated annealing algorithm, which can effectively compensate for the deficiencies of both sides. The core idea of the GSA algorithm is to introduce a simulated annealing operation after the genetic operation step, so that the genetic algorithm dominates the global search and the simulated annealing algorithm dominates the local optimization process. Crossover and mutation in genetic algorithms do not have any goal and direction as the operation to guide the evolution of the population. The annealing operation in simulated annealing will provide a targeted screening guide for the evolution of the individual population.

Aiming at the shortcomings of genetic algorithm and simulated annealing algorithms, there is still some room for improvement to improve the efficiency and accuracy of the algorithm.

*Improve Crossover and Mutation Probability*. According to the above analysis, the crossover probability *P*_*c*_ and mutation probability *P*_*m*_ have a decisive influence on the efficiency of the genetic algorithm. The crossover probability determines the diversity, and the mutation probability determines the ability to jump out of the local optimum. But general genetic algorithms usually set the two to be constant, and it is difficult to debug to the optimal value. In this regard, this study adopts the concentration and dispersion degree of fitness in the population to set the crossover mutation probability of adaptive change:

(7) $$\begin{array}{c} P_{c}=\left\{\begin{array}{cc} 2k_{1}\frac{\arcsin\left(f_{a}/f_{m}\right)}{\pi },\; & \arcsin\left(\frac{f_{a}}{f_{m}}\right)<\pi /6,\\ k_{1}\left(1-\frac{2\;\arcsin\left(f_{a}/f_{m}\right)}{\pi }\right), & \text{others,} \end{array}\right)\\ P_{m}=\left\{\begin{array}{cc} k_{2}\left(1-\frac{2\;\arcsin\left(f_{a}/f_{m}\right)}{\pi }\right), & \arcsin\left(\frac{f_{a}}{f_{m}}\right)<\pi /6,\\ 2k_{2}\frac{\arcsin\left(f_{a}/f_{m}\right)}{\pi }, & \text{others}. \end{array}\right) \end{array}$$

This method can generate a more diverse and rich population of individuals during the crossover process, while retaining the excellent genetic inheritance and strengthening the global search ability. Self-adaptation increases the mutation probability at the beginning and end of the algorithm, accelerates the convergence speed of the algorithm, and gives the algorithm a stronger ability to jump out of the local optimum.

*Improve Metropolis Criterion*. The simulated annealing algorithm has excellent global optimization ability, but the computational proficiency is slow, and the judgment criteria usually used are based on standard criteria. This kind of comparison and screening of new populations in a fixed way can easily cause other better solutions with the same convergence ability to be ignored in the process of global optimization, resulting in local convergence. Here, an improved Metropolis criterion is used to optimize the judgment conditions of the old individual and the new individual. The improvement criterion is determined as follows when comparing the old and new populations with the genetic algorithm:

(8) $$\begin{array}{c} P=\exp\left(\frac{f\left(x_{o}\left(j\right)\right)-f\left(x_{n}\left(j\right)\right)}{kT}\right). \end{array}$$

In the process of judging the old and new populations, the poor new population individuals are modified and improved, their fitness values are improved, and they are accepted as offspring with probability *P*. By adopting this method, the genetic algorithm can be linked with the simulated annealing algorithm, the population diversity and the global optimization ability of the simulated annealing algorithm can be improved, and the dilemma of falling into the local optimum can be avoided. The structure of IGSA is illustrated in Figure 3.

### 3.5. Evaluation of PDCA Nursing in Asthma Treatment with IGSA-BP

The effect evaluation process of the PDCA nursing model based on the IGSA-BP network in the treatment of childhood asthma is shown in Figure 4.

The specific treatment effect evaluation steps are as follows: (1) collect data to form the training set and test set of the BP algorithm. (2) Randomly initialize the weights and thresholds, and use the IGSA algorithm to output the optimal solution of the algorithm. After decoding, the initial connection weights and thresholds of each neuron in the neural network are obtained. (3) Import these connection weights and thresholds into the BP network to obtain the optimized BP neural network. (4) Using the data obtained in the first part again, the BP network is trained and learned, and the network effect is verified through the test set.

## 4. Experiment Result

### 4.1. Dataset

This work uses two self-made datasets to evaluate the effect of the electronic health PDCA nursing model in the treatment of childhood asthma such as CAA and CAB. Each dataset contains different numbers of samples. The specific information is listed in Table 2. The input of each sample data is 8 efficacy indicators, the specific indicators are listed in Table 3, and the corresponding label is the efficacy classification, which is divided into 10 efficacy levels. The evaluation metrics used in this work are precision and recall.

### 4.2. Evaluation on Network Training

In neural networks, the convergence of the network is a very important indicator. Only when the network reaches a state of convergence on the training set, the most basic correctness of the network can be proved. To evaluate the convergence of the network designed in this work, the loss change of the network during training is evaluated. The experimental results are shown in Figure 5.

It can be seen that as the training progresses, the loss of the network decreases sharply, then decreases slowly, and finally stabilizes. This shows that the network finally reaches the convergence state and also proves the correctness of the network designed in this work.

### 4.3. Comparison with Other Methods

To verify the validity of the IGSA-BP network for evaluating the effect of the e-health PDCA care model in the treatment of childhood asthma, this section compares the designed method with other methods. Other methods involved include logistic regression (LR), decision tree (DT), and SVM. The experimental results are listed in Table 4 and comparison of tuned parameters is listed in Table 5.

It is obvious that the method designed in this work can achieve the best performance. Compared with the best performing SVM method in the table, IGSA-BP can achieve 2.8% precision improvement and 2.4% recall improvement on CAA dataset, and 3.5% precision improvement and 3.8% recall improvement on CAB dataset. This further verifies the correctness and effectiveness of the method designed in this work.

### 4.4. Evaluation on IGSA-BP

As mentioned earlier, the IGSA-BP algorithm designed in this work is firstly to combine the genetic algorithm (GA) with the simulated annealing algorithm (SA), then improve it, and finally combine it with the BP network. To verify the effectiveness of this strategy, different comparative experiments are conducted in this section. First, in order to verify that introducing SA into this network can improve network performance and compare the performance with and without SA, and the results are illustrated in Figure 6.

It can be seen that when the SA algorithm is introduced, IGSA-BP can achieve 2.4% precision improvement and 2.9% recall improvement on the CAA dataset, and 2.6% precision improvement and 2.1% recall improvement on the CAB dataset. This further verifies the correctness and effectiveness of using GA.

To further verify that the improved genetic simulated annealing algorithm can improve the network performance, another set of comparative experiments was conducted. This work compares the efficacy evaluation performance when using GSA-BP and IGSA-BP, and the experimental results are shown in Figure 7.

It can be seen that when the improvement strategy is introduced, IGSA-BP can achieve 1.0% precision improvement and 0.7% recall improvement on the CAA dataset, and 1.2% precision improvement and 1.3% recall improvement on the CAB dataset. This further verifies the correctness and effectiveness of the improvement strategy on IGSA.

## 5. Conclusion

In this study, IGSA is utilized to optimize the BP network to evaluate the effect of the electronic health PDCA nursing model in the treatment of childhood asthma. Aiming at the problems of slow training convergence speed and falling into local optimum, this work adopts combination of GA and SA. Only the combined method is further improved to optimize initial weights as well as thresholds. Finally, an evaluation model of children's asthma treatment effect was built, and the feasibility and reliability of the method were verified by simulation analysis. The main work content and research results are as follows: (1) in view of the problems that the results of the BP network are easily affected by initial weights as well as thresholds, and convergence is slow and easy to fall into local optimization, this work proposes to optimize BP network by using GA and SA. Finally, the effect of the electronic health PDCA nursing model in the treatment of children's asthma was evaluated. (2) Analyze and summarize the principles of GA and SA algorithms and their respective advantages and disadvantages, and design an IGSA algorithm. By improving crossover and mutation probability, an adaptive adjustment in genetic processes can speed up algorithm convergence speed. By improving the Metropolis criterion, the global optimization ability is improved. On the basis of the BP network, the evaluation model of the electronic health PDCA nursing mode based on IGSA-BP in the treatment of children's asthma was designed.

## Figures and Tables

**Figure 1:** The structure of BP.

**Figure 2:** Genetic algorithm flowchart.

**Figure 3:** The structure of IGSA.

**Figure 4:** Schematic diagram of IGSA-BP treatment effect evaluation.

**Figure 5:** The training loss on (a) CAA and (b) CAB.

**Figure 6:** Evaluation on SA.

**Figure 7:** Comparison of (a) GSA-BP and (b) IGSA-BP.

**Table 1:** Comparison of literature.

Aim and reference	Problem-solving technique	Application	Result
Individualized interventional pain management technique in early stage of cancer pain: a desirable protocol for improving quality of life (J). [16]	PDCA	Education of nursing	Improved

Prospective, observational study of pain and analgesic prescribing in medical oncology outpatients with breast, colorectal, lung, or prostate cancer (J). [17]	PDCA	Blood glucose testing	Improved

Morphine as the first drug for the treatment of cancer pain (J). [18]	PDCA	In ICU for reducing the rate of catheter-related blood infection.	Good

Models of palliative care delivery in the United States (J). [19]	FOCUS-PDCA	Solving multifaceted and complex clinical nursing quality problems	Good

Minnesota rural palliative care initiative: building palliative care capacity in rural Minnesota (J). [20]	PDCA	Severe traumatic brain injury	Good

Analysis of PDCA circulation guidance in the whole-course diabetes health education (J). [21]	PDCA	Diabetes-health-education-research	Remarkable

Effect of follow-up management based on PDCA circulation combined with PIO in diabetic patients complicated with non-alcoholic fatty liver (J). [22]	PDCA	Management of T2DM patients with NAFLD	Improved

Effect evaluation of PDCA cycle on postoperative rehabilitation health education among patients with lumbar minimally invasive surgery (J). [23]	PDCA	Postoperative rehabilitation health education	Improved

Effects of PDCA circulation health education on children's asthma control level (J). [24]	PDCA	Control of childhood asthma	Good

Effect of PDCA nursing mode on angina pectoris and quality of life after discharge in patients with myocardial infarction (J). [25]	PDCA	Patients with myocardial infarction	Improved

Application of PDCA nursing mode in the course of nursing the patients with pernicious placenta previa (J). [26]	PDCA	Implemented nursing intervention	Improved

Effect of health education in occupational population with high-blood pressure based on PDCA model (J). [27]	PDCA	Blood pressure level	Good

Effects of PDCA circulation health education on children's asthma control level (J). [28]	PDCA	Implementation of gastroenterology health education	Satisfactory

Application of PDCA circulation theory in buccal clinical nursing teaching (J). [29]	PDCA	Oral and gynecology clinical teaching	Good

Using PDCA cycle to improve the quality of nursing records (J). [30]	PDCA	Nursing record quality management	Improved

The value analysis of PDCA cycle in the application of management of the quality of emergency care (J). [31]	PDCA	Emergency department	Improved

Effect of PDCA circulation on improving quality of nursing quality in outpatient operation room (J). [32]	PDCA	Oral diagnosis and nursing management	Good

**Table 2:** The detailed information of CAA and CAB.

Dataset	Training set	Test set
CAA	589	206
CAB	817	398

**Table 3:** The detailed efficacy indicators.

Item	Index
*X*_1_	Relief of wheezing symptoms
*X*_2_	Relief of shortness of breath symptoms
*X*_3_	Relief of hypoxia symptoms
*X*_4_	Relief of chest tightness symptoms
*X*_5_	Relief of lung function symptoms
*X*_6_	Exhaled nitric oxide concentration
*X*_7_	Induces the concentration of eosinophils
*X*_8_	Peripheral blood eosinophil concentration

**Table 4:** Comparison with other methods.

Method	CAA		CAB	
	Precision	Recall	Precision	Recall
LR	83.7	81.1	85.9	82.6
DT	87.2	84.6	89.5	86.7
SVM	91.7	89.8	93.2	91.1
IGSA-BP	94.5	92.2	96.7	94.9

**Table 5:** Comparison of tuned parameters for AI algorithms.

Sr. No.	Ai algorithm	Tuned parameters
1	Logistic regression	Penalty-l2, tol-0.0001, C-(0.1–1.0), max_iter-(50–100)
2	Decision tree	Max_depth-(100–200), min_samples_split-2, min_samples_leaf-1
3	Support vector machine	n-estimators, max_depth-(100–200), min_samples_split-2
4	IGSA-BP	n_iterations-(100–200), step_size-(0.1–1.0), min-0.1, max-0.1

## Data Availability

The datasets used during the current study are available from the corresponding author on reasonable request.
